# Antilingula as a Surgical Reference Point for Vertical Ramus Osteotomy

**DOI:** 10.1155/2021/5585297

**Published:** 2021-04-20

**Authors:** Han-Sheng Chen, Ying-Sheng Chen, I-Ling Lin, Chun-Feng Chen

**Affiliations:** ^1^Dental Department, Kaohsiung Municipal Siaogang Hospital, Kaohsiung, Taiwan; ^2^Dental Department, Taipei Medical University-Shuang Ho Hospital, Taipei, Taiwan; ^3^Department of Medical Laboratory Science and Biotechnology, College of Health Sciences, Kaohsiung Medical University, Kaohsiung, Taiwan; ^4^Department of Oral and Maxillofacial Surgery, Kaohsiung Veterans General Hospital, Kaohsiung, Taiwan; ^5^School of Dentistry, College of Dental Medicine, Kaohsiung Medical University, Kaohsiung, Taiwan; ^6^Department of Dental Technology, Shu-Zen Junior College of Medicine and Management, Kaohsiung, Taiwan

## Abstract

**Purpose:**

This study investigated the antilingula and its related landmarks, the mandibular rami, by using cone-beam computed tomography (CBCT).

**Methods:**

CBCT images of 37 patients (74 sides of the mandibular ramus) were collected. The landmarks of antilingula (AntiL), anterior ramus (A), posterior ramus (P), superior ramus (S), and inferior ramus (I) were identified. The distances (A-AntiL, P-AntiL, S-AntiL, and I-AntiL) were statistically evaluated according to gender, side (right and left), and skeletal patterns.

**Results:**

The distance from the antilingula to the anterior (A-AntiL) border of the ramus was significantly longer on the right side (14.69 mm) than on the left side (13.97 mm). Male patients had longer AntiL-P, AntiL-I, and S-I distances (18.96, 40.07, and 54.94 mm, respectively) than did female patients (16.66, 35, and 47.54 mm, respectively). Regarding skeletal patterns, the classes can be ordered as follows in terms of the measurements: class III>class II>class I. However, the differences between the classes were nonsignificant. Pearson correlation analysis revealed that gender and S-I distance were strongly correlated (*r* = 0.667); specifically, male patients had a longer S-I distance. A-AntiL and A-P also exhibited a strong correlation (*r* = 0.796).

**Conclusion:**

Antilingula-related distances did not differ between skeletal patterns. Among antilingula-related variables, A-AntiL could serve as a favorable measuring point during operation.

## 1. Introduction

Most patients with class III malocclusions seek corrective treatment to improve their appearance, social confidence, and interpersonal relationships, among other reasons. Sagittal split ramus osteotomy (SSRO) and intraoral vertical ramus osteotomy (IVRO) are the most commonly adopted surgical techniques for treating mandibular protrusions. SSRO involves making a horizontal cut from above the mandibular foramen on the inner surface of the ramus, specifically at or above the lingula, continuing forward and outward to the external oblique ridge and then to the buccal side of the molar. In SSRO, the mandible is divided into two segments: lingual and buccal parts (distal and proximal segments). By contrast, IVRO involves making vertical or oblique cut behind the mandibular foramen on the ramus buccal side. In IVRO, the mandible is divided into two segments: anterior and posterior parts (distal and proximal segments).

Identifying and accessing the lingula in IVRO technique is difficult from buccal side of ramus. To resolve this difficulty, Aziz et al. [1] revealed that the antilingula is an acceptable landmark for the safe placement of IVRO to prevent damage to the inferior alveolar nerve in the mandibular foramen. Such damage can lead to complications associated with sensory disorders, particularly in the lower lip [2–4]. However, Monnazzi et al. [5] reported no statistically significant correlation between the mandibular foramen entrance and the antilingula position. The antilingula is a small bony protuberance on the buccal surface of the mandibular ramus; it is not an independent point of protuberance and is thus sometimes difficult to identify. Moreover, whether the antilingula differs with respect to the three classes of skeletal patterns (class I, class II, and class III) is critical for surgeons; however, this question has not been thoroughly investigated by researchers. Accordingly, the present study investigated the differences in the position of the antilingula between patients with skeletal class I, class II, and class III malocclusions and determined their related variables.

## 2. Materials and Methods

This study obtained cone-beam computed tomography (CBCT; NewTom VGi EVO, Imola, Italy) images of 37 patients (15 men and 22 women)—with a total of 74 face sides—from the Department of Dentistry of Kaohsiung Medical University Hospital. These images were used for analysis. The exposure parameters were as follows: tube voltage, 110 kV; tube current, 4.59 mA; and slice thickness, 0.2 mm. Patients with the following characteristics were excluded from the sample: (1) congenital craniofacial symptoms, (2) orthognathic surgery, or (3) facial bone injury. The reference plane for the 3D images, namely, the Frankfort horizontal plane, was defined as the plane connecting the lower margin of the right orbit and the uppermost points of the external auditory meatus on each side. For consistency and replicability, this study calibrated all patients' CBCT images with respect to the following positions: (1) the sagittal plane was positioned at the orbit to divide the skull evenly into the right and left parts, (2) the horizontal plane was positioned parallel to the Frankfort horizontal plane, and (3) the coronal plane was positioned perpendicular to the aforementioned planes.

The collected images (DICOM format) were imported into RadiAntViewer (version 4.6.9, Medixant, Poznan, Poland), after which RadiAntViewer's 3D image reconstruction function was used to extract and reconstruct 3D images of the mandibular ramus. The reconstructed images were then used to examine the antilingula (AntiL) on the buccal surface of the mandibular ramus. Each patient's gender and skeletal pattern were recorded, and images of both sides of the patient's mandible were taken. Patients were categorized into three groups according to their skeletal patterns: class I (0° < A point–nasion–B point angle [ANB] < 4°), class II (ANB ≥ 4°), and class III (ANB ≤ 0°). The axis of ramus was set as a tangent line passing through the posteriormost borders of the condyle and ramus (Figure 1). Through the AntiL point, a line parallel to the ramus axis and another line perpendicular to this axis were considered. This study measured the distances from the antilingula to the anterior (A-AntiL) and posterior (P-AntiL) borders of the ramus as well as those from the antilingula to the superior (S-AntiL) and inferior (I-AntiL) borders of the ramus. The study also determined the relative positions of the antilingula on the path between the anterior and posterior (A-P) borders and the path between the superior and inferior (S-I) borders.

This study also investigated the differences in A-AntiL, P-AntiL, S-AntiL, and I-AntiL between the left and right sides of the mandible, between female and male patients and between the three skeletal patterns. Moreover, the correlation of these distances with sex and skeletal patterns was investigated. IBM SPSS 20 (SPSS Inc., Chicago, IL, USA) was used for statistical analysis, and a *P* value of 0.05 was considered statistically significant. One-way analysis of variance was used to examine the differences between the three skeletal pattern classes, followed by post hoc analysis using the Tukey method. The Pearson correlation analysis was used to determine the correlations between variables (gender, skeletal patterns (classes I, II, III), and AntiL-related distances). Different facial skeletal patterns may differ significantly in terms of the anatomical structures of the mandible. Therefore, the null hypothesis was that the AntiL-related distances would not differ between the three skeletal patterns. The strengths of the correlations were determined as follows: very weak (0–0.19), weak (0.20–0.39), moderate (0.40–0.59), strong (0.60–0.79), and very strong (0.80–1.0). This retrospective study was approved by the Institutional Review Board of Kaohsiung Medical University Hospital (KMUH-IRB-20160066).

## 3. Results

As presented in Table 1, A-AntiL was significantly longer on the right side of the mandible (14.69 mm) than it was on the left side (13.97 mm). The other linear distances (P-AntiL, A-P, S-AntiL, I-AntiL, and S-I) did not differ significantly between the sides of the mandible. Overall, the antilingula was located along the A-P border at the point extending 45% backward from the anterior border of the ramus and along the S-I border at the point extending 27% downward from the superior border of the ramus. As listed in Table 2, male patients had longer AntiL-P, AntiL-I, and S-I (18.96, 40.07, and 54.94 mm, respectively) than did female patients (16.66, 35, and 47.54 mm, respectively).

As shown in Table 2, male patients' antilingula was located along the A-P border at the point extending 44% backward from the anterior border of the ramus and along the S-I border at the point extending 27% downward from the upper border. Female patients' antilingula was located along the A-P border at the point extending 45% backward from the anterior border and along the S-I border at the point extending 26% downward from the upper border. Accordingly, the location of male patients' antilingula was slightly ahead of and below that of female patients' antilingula.

Regarding the skeletal patterns (Table 3), the three classes can be ordered as follows in terms of the measurements for the A-P and S-I distances: class III>class II>class I. However, the differences between the classes were nonsignificant. Therefore, the null hypothesis was accepted. According to the Pearson correlation analysis (Table 4), gender and S-I were strongly correlated (*r* = 0.667); specifically, male patients had a longer S-I. A-AntiL and A-P were strongly correlated (*r* = 0.796). Moreover, S-AntiL and S-I were strongly correlated (*r* = 0.617). I-AntiL and S-I were very strongly correlated (*r* = 0.831).

## 4. Discussion

The term “antilingula” was introduced in the study by Levine and Topazian [6] and was used a reference point for inverted-L osteotomy; according to Levine and Topazia, the antilingula is formed by the inferior alveolar nerve entering the mandibular ramus, which causes a protuberance on the outer surface of the bone. However, other researchers have proposed different views. Reitzik et al. [7] proposed that the protuberance on the outer surface of the mandibular ramus is the attachment point for the masseter muscle; the researchers also described the protuberance as a masseteric apical bump. Furthermore, subsequent studies [8–10] on humans and other mammals have confirmed that the protuberance on the outer surface of the mandibular ramus is the attachment point for the deep head of the masseter muscle. The pattern of attachment of the masseter muscle on the mandibular ramus and the force of the masseter muscle can both affect the formation of the antilingula and the size of the protuberant area. However, the antilingula is not always noticeable or identifiable on the mandible.

Previous studies [11–13] have demonstrated the relationship between the position of the antilingula and that of the lingula and mandibular foramen. Scholars [13–15] have suggested that the position of the antilingula—which can be seen during operation—exhibited a stable relationship with the position of the mandibular foramen. Accordingly, these scholars [13–15] have recommended that the position of the bone cut in IVRO could be determined with reference to the position of the antilingula; specifically, the osteotomy line should be placed behind the antilingula to prevent damage to the inferior alveolar nerve. By contrast, the relative position of the antilingula to the lingual and mandibular foramen is characterized by a high degree of uncertainty. Studies [16, 17] have indicated that the position of the antilingula is not fixed relative to the position of the lingula and mandibular foramen; therefore, the use of the antilingula as the surgical reference point for IVRO has been discouraged. Nevertheless, Aziz et al. [1] reported that in most cases, the lingula is located inferior to and behind the antilingula. Pogrel et al. [17] also reported a 68.3% probability of the lingula being located inferior to and behind the antilingula, with the average distance between them being 5.39 mm. Furthermore, Park et al. [13] revealed that on average, the lingula was located 4.19 mm backward and 0.54 mm upward relative to the antilingula. The mandibular foramen was located 4.98 mm backward and 6.95 mm downward relative to the antilingula.

The aforementioned research findings [1, 13–17] are all consistent in that the osteotomy line in IVRO should be placed behind the antilingula to prevent damage to the inferior alveolar nerve. Park et al. [13] reported that to completely avoid the inferior alveolar nerve in IVRO, the osteotomy line should be in the posterior region at a point located at 29% of the total horizontal length of the ramus. However, simply using the antilingula as the primary reference point for the osteotomy line could increase the possibility of damage to the inferior alveolar neurovascular bundle. Therefore, locating the positions of the lingula and mandibular foramen on the anterior-posterior and superior-inferior dimensions of the mandibular ramus may be the only approach to determining the safe osteotomy line in IVRO. Because a complete anatomical structure measurement for IVRO has yet to be developed, the position of the antilingula cannot serve as the absolute reference point for such surgical operations.

Hosapatna et al. [18] studied 50 dry mandibles and observed that the antilingula was located on the right side of 25 of the mandibles and on the left side of 28 of the mandibles. Hsiao et al. [19] reported the bilateral presence of the antilingula in 67.8% of those studied. The present study revealed diverse antilingula patterns; specifically, the antilingula can manifest as a marked protuberance or a plateau-shaped protuberant area without a single point of protuberance, which can result in misjudgment. In particular, cases of plateau-shaped protuberant areas are not rare, and any resulting misjudgment can damage the neurovascular bundle. Accordingly, the present study selected patients who exhibited a single point of protuberance on both the left and right sides of the mandible for observation and comparison; they were selected because the antilingula can be adopted as the reference point for surgery only in these patients. According to the study results, the left and right sides of the mandible did not differ significantly with respect to A-P or S-I distances; this finding signifies that the lengths of the mandibular rami on the left and right sides were similar in these patients, which can facilitate a relatively consistent determination of bone cut position regardless of the side of the mandible, thus increasing the safety of surgical operations.

Male patients' A-P and S-I distances were both greater than those of female patients, a finding that is consistent with the clinical observation that male mandibles tend to be larger than female mandibles. Moreover, male patients' AntiL-P, AntiL-I, and S-I distances (18.96, 40.07, and 54.94 mm, respectively) were significantly longer than those of female patients (16.66, 35, and 47.54 mm, respectively). Male patients' antilingula was located along the A-P border at the point extending 44% backward from the anterior border and along the S-I border at the point extending 27% downward from the superior border of the mandibular ramus. Female patients' antilingula was located along the A-P border at the point extending 45% backward from the anterior border and along the S-I border at the point extending 26% downward from the superior border of the mandibular ramus. Accordingly, male patients' antilingula was located slightly ahead of and below that of female patients. However, whether male patients' mandibular foramen is*—*similar to their antilingula*—*located at a similar position to that of female patients requires further research; answering this question can prevent misjudgment and damage to the neurovascular bundle in surgical operations.

Regarding the skeletal patterns, the three classes can be ordered as follows in terms of their A-P and S-I distances: class III>class II>class I. This finding is consistent with the clinical observation that class III patients had noticeably larger mandibles. Nevertheless, the different skeletal patterns had nonsignificant differences with respect to various relevant measurements. Gender exhibited a more significant correlation with S-I than it did with A-P. Therefore, the male sex had a stronger correlation with ramus height than it did with ramus width.

The significant relationships of P-AntiL involved more factors (gender, skeletal pattern, A-P, S-AntiL, I-AntiL, and S-I) than did those of A-AntiL, which involved only the factors A-P and I-AntiL. However, using AntiL-P to determine the position of the antilingula is difficult in clinical surgery because the posterior border of the mandible ramus is usually curved and inward. Measuring tools used in surgical operations cannot be bent for precise measurement of the posterior border of the ramus; this difficulty leads to high measurement errors. Therefore, measurements should be performed from the anterior border of the ramus (i.e., A-AntiL) to reduce measurement errors.

The significant relationships of I-AntiL involved more factors (sex, A-AntiL, AntiL-P, A-P, and S-I) than did those of S-AntiL, which involved only the factors P-AntiL and S-I. In clinical surgery, the sigmoid notch is used to determine the position of the antilingula. However, because the sigmoid notch is semicircular, the measuring tool can slip during operation, which can lead to an inaccurate determination of the antilingula position relative to the sigmoid notch. By contrast, the mandibular inferior border has a relatively flat shape and can thus facilitate relatively stable measurement. Accordingly, compared with S-AntiL, using I-AntiL to determine the position of the antilingula is more practicable and results in fewer errors. Considering surgical accessibility and convenience, A-AntiL is a more favorable measuring point than I-AntiL.

## 5. Conclusion

The antilingula cannot be the sole reference point for IVRO. Antilingual distances do not differ according to skeletal patterns. Among antilingula-related variables, A-AntiL can serve as a favorable measuring point during operation.

## Figures and Tables

**Figure 1:** Red point: AntiL (antilingula); S: superior point of ramus; I: inferior point of ramus; A: anterior point of ramus; P: posterior point of ramus. Green line: axis of ramus (a tangent line passing through most posterior borders of condyle and ramus). Blue line: a line through AntiL and parallel to green line. Yellow line: a line through AntiL and perpendicular to blue line.

**Table 1:** Antilingula-related distances with their hemiarch comparisons.

Variables	Total patients (*n* = 37)		Right side		Left side		Right/left comparison	
	Mean	SD	Mean	SD	Mean	SD	*P* value	Significant
A-AntiL	14.32	2.62	14.69	2.61	13.97	2.61	0.030	Right>left
P-AntiL	17.59	2.12	17.47	2.14	17.72	2.13	0.483	─
A-P	31.92	3.51	32.2	3.50	31.7	3.55	0.157	─
S-AntiL	13.48	3.07	13.33	2.89	13.63	3.27	0.455	─
I-AntiL	37.06	4.33	37.54	4.16	36.57	4.48	0.064	─
S-I	50.54	5.49	50.9	5.15	50.2	5.85	0.224	─

AntiL: antilingula; A: anterior ramus; P: posterior ramus; S: superior ramus; I: inferior ramus. *n*: number of patient; significant: *P* < 0.05; ─: not significant.

**Table 2:** Antilingula-related distances with their gender comparisons.

Variables	Male (*n* = 30)		Female (*n* = 44)		Gender comparison	
	Mean	SD	Mean	SD	*P* value	Significant
A-AntiL	14.92	3.10	13.90	2.18	0.540	─
P-AntiL	18.96	1.98	16.66	1.68	0.021	Male>female
A-P	33.90	3.86	30.57	2.50	0.078	─
S-AntiL	14.87	3.17	12.53	2.63	0.408	─
I-AntiL	40.07	3.16	35.00	3.79	0.002	Male>female
S-I	54.94	4.25	47.54	4.03	0.001	Male>female

AntiL: antilingula; A: anterior ramus; P: posterior ramus; S: superior ramus; I: inferior ramus. *n*: number of side; significant: *P* < 0.05; ─: not significant.

**Table 3:** Antilingula-related distances with their skeletal patterns.

Variables	Class I (*n* = 28)		Class II (*n* = 24)		Class III (*n* = 22)		Interclass comparison		
	Mean	SD	Mean	SD	Mean	SD	*F* value	*P* value	Significant
A-AntiL	14.03	2.43	14.04	2.39	14.98	3.07	1.005	0.371	─
P-AntiL	16.98	2.19	17.67	1.98	18.29	2.05	2.485	0.091	─
A-P	31.00	3.28	31.73	2.62	33.30	4.29	2.814	0.067	─
S-AntiL	13.01	2.71	13.27	3.29	14.30	3.22	1.175	0.315	─
I-AntiL	36.58	4.29	36.45	3.79	38.32	4.82	1.357	0.264	─
S-I	49.60	4.51	49.74	5.13	52.62	6.57	2.338	0.104	─

AntiL: antilingula; A: anterior ramus; P: posterior ramus; S: superior ramus; I: inferior ramus. *n*: number of side; significant: *P* < 0.05; ─: not significant.

**Table 4:** Gender and skeletal patterns of antilingula-related distances in the Pearson test.

Variables	Gender	Skeletal	A-AntiL	P-AntiL	A-P	S-AntiL	I-AntiL	S-I
Gender	1	0.418^∗^	0.192	0.534^∗^	0.468^∗^	0.376^∗^	0.579^∗^	0.667^∗^
Skeletal	0.418^∗^	1	0.143	0.256^∗^	0.265^∗^	0.169	0.158	0.219
A-AntiL	0.192	0.143	1	0.084	0.796^∗^	-0.135	0.280^∗^	0.145
P-AntiL	0.534^∗^	0.256^∗^	0.084	1	0.670^∗^	0.255^∗^	0.297^∗^	0.377^∗^
A-P	0.468^∗^	0.265^∗^	0.796^∗^	0.670^∗^	1	0.054	0.387^∗^	0.336^∗^
S-AntiL	0.376^∗^	0.169	-0.135	0.255^∗^	0.054	1	0.075	0.617^∗^
I-AntiL	0.579^∗^	0.158	0.280^∗^	0.297^∗^	0.387^∗^	0.075	1	0.831^∗^
S-I	0.667^∗^	0.219	0.145	0.377^∗^	0.336^∗^	0.617^∗^	0.831^∗^	1

AntiL: antilingula; A: anterior ramus; P: posterior ramus; S: superior ramus; I: inferior ramus. Significant: *P* < 0.05; ─: not significant.

## Data Availability

The data used to support the findings of this study are included within the article.
